# Emodin Interferes With AKT1-Mediated DNA Damage and Decreases Resistance of Breast Cancer Cells to Doxorubicin

**DOI:** 10.3389/fonc.2020.588533

**Published:** 2021-02-09

**Authors:** Bo Li, Xin Zhao, Lei Zhang, Wen Cheng

**Affiliations:** ^1^ Department of Ultrasound, Harbin Medical University Cancer Hospital, Harbin, China; ^2^ Department of Orthopedics, The Second Affiliated Hospital of Harbin Medical University, Harbin, China; ^3^ Department of Ultrasound, The Second Affiliated Hospital of Harbin Medical University, Harbin, China

**Keywords:** emodin, AKT1, bioinformatics, DNA repair, breast cancer

## Abstract

Doxorubicin (DOX) is a cytotoxic drug used for the treatment of breast cancer (BC). However, the rapid emergence of resistance toward doxorubicin threatens its clinical application, thus the need for combination therapy. Here, we interrogate the role of Emodin, a chemical compound with tumor inhibitory properties, in the resistance of BC to Doxorubicin. We first evaluated the efficacy of Emodin in the treatment of BC cells. We then used γH2A to examine doxorubicin-induced DNA damage in BC cells, with or without Emodin. Data from CCK-8, flow cytometry, and tumor xenograft assays showed that Emodin suppresses the growth of BC cells. Further, we demonstrated that Emodin enhances γH2A levels in BC cells. Moreover, bioinformatics analysis and western blot assays indicated that Emodin down-regulates the AKT1 expression, and marginally decreases the levels of DNA damage proteins (XRCC1, PARP1, and RAD51) as well as increased p53 expression in BC cells. Taken together, our data demonstrates that Emodin affects cell proliferation, and DNA damage pathways in BC cells, thus increasing the sensitivity of BC cells to doxorubicin. Besides, we confirmed that Emodin confers sensitization of BC to doxorubicin through AKT1-mediated DNA.

## Introduction

Breast cancer (BC) is one of the most common types of cancer in females. The last two decades has seen a steady rise in BC cases in China (1, 2). BC is classified according to the hormone receptors: progesterone receptor (PR), estrogen receptor (ER), or human epidermal growth factor receptor 2 (HER2), which define diverse clinical outcomes and responses to treatment. Triple-negative breast cancer (TNBC), accounts for 15% to 20% of all the BCs and is often associated with poor survival upon disease relapse (3–5). The deficiency of the three receptors coupled with the emerging drug resistance present a major challenge in developing precise drugs for the treatment of BC (6, 7). Whereas recent advances have reduced chemotherapy resistance (8), there is still a need for a more effective drug regimen in BC.

Cytotoxic drugs often induce DNA damage and cancer cell apoptosis leading to death (9). Doxorubicin, a known is a commonly chemotherapeutic for BC (10, 11), kills cancer cells by inducing DNA-crosslinking damage, which if not properly repaired, leads to double strand breaks and ultimate cellular death (12, 13). Evidence showed that doxorubicin had anti-cancer effect at a higher concentration which produce cardiotoxicity (14). Prolonged use of doxorubicin chemotherapy with long term leads to drug resistant which could be overcome by combination treatment with other agents (15, 16). Therefore, it is urgent to find some possibilities agents to increase its efficacy on BC cells with doxorubicin.

Emodin (6-methyl-1, 3, 8-trihydroxyanthraquinone, C15H10O5), an agent mainly isolated from Rheum Palmatum and used as a Chinese medicinal herb, has many pharmacological benefits (17, 18). Emodin has liver protective properties (19), anti-inflammatory (20, 21), and anti-viral effects (22). It is also associated with immune regulation (23), promotion of gastrointestinal motility (24), as well as antioxidant properties (25).

AKT1 is a key protein that regulates many apoptotic pathways in response to DNA damage (26). AKT1 also plays a major role in chemotherapy and drug resistance (27). Other studies have shown that Emodin could disrupt DNA damage response in cervical as well as oral squamous carcinoma cell lines (13). However, the relationship between Emodin, AKT1 and DNA damage in BC is still unclear.

Here, we explored whether Emodin improves the effect of doxorubicin in BC and investigated potential mechanisms. We reveal the beneficial roles of Emodin in reducing drug- resistance in BC as well as provide a new drug regimen for the treatment of BC.

## Materials and Methods

### Cell Culture

Breast cancer (MDA-MB-231 as well as MCF-7) cell lines were attained from the Cell Bank of Chinese Academy of Sciences (Shanghai, China). The BC cells were cultured in 1640 (Invitrogen, USA) with 10% FBS (fetal bovine serum, Invitrogen, USA), 100 U/ml penicillin, as well as 50 μg/ml streptomycin (Invitrogen, USA). The cells were kept at a 37°C incubator with proper humidity and 5% CO_2_.

### Real-Time PCR

RNA was isolated form the cells and tissue using the TRIzol reagent (Invitrogen, USA). The reaction used Power SYBR Green PCR master Mix (Life Technologies; Thermo Fisher Scientific, USA) with the following primer pairs;

AKT1-F: 5’- GCAGCAACTGTACTCGTCG-3’;
AKT1-R: 5’- GACTCCACGCACTCAAGGTA-3’
Actin-F: 5’-CAATGTACTGTTGCTATACCAGGC-3’;
Actin-R: 5’-CATCCTTAATTGTCACGACACGAT-3’.

### AKT1-siRNA and Plasmid Transfection

AKT1 overexpression plasmid or AKT1 siRNA (small interference RNA) was constructed by RiboBio. Breast cancer cells were transfected with siRNA or plasmid using RiboFECT™CP Transfection kit (C10511-05, RiboBio, Guangzhou, China) following the manufacturer’s protocol.

### Western Blot

We lysed the cells using the RIPA buffer with a protein inhibitor (Roche, Switzerland; 1:100), and the concentration of the proteins was estimated using the BCA kit (Beyotime Biotechnology, Shanghai, China). The proteins were then resolved in a 12.5% SDS-PAGE (Beyotime Biotechnology, Shanghai, China) and transferred to a cellulose acetate membrane (Thermo Scientific, USA). The blot was developed by blocking in 5% non-fat milk for 2 h at RT (room temperature), and then incubated with primary antibodies against β-Actin, XRCC1, PARP1 or AKT1 (Cell Signaling Technology, USA), and p53, RAD51 (Abcam, UK), overnight. The blots were washed with PBST (500 ml PBS+200 µl TWEEN 20) three times and then incubated with either rabbit or mouse secondary antibodies (CST, USA) at room temperature for 1 h. The blots were detected using enhanced chemiluminescence (ECL) reagents (GE, USA).

### Cell Viability Assays Using Cell Counting Kit-8 (CCK-8)

MCF-7 and MDA-MB-231 cells were treated with Emodin. Cells (5 × 10^3^) were sowed into 96-well plates for 48 h and then the cell growth was determined using the CCK-8 (Dojindo, Japan).

### γH2A Immunofluorescence Staining

The MCF-7 and MDA-MB-231 cells were mounted on cover slips for 24 h with a density of 50% to 60% and then treated with Doxorubicin, Emodin, or Doxorubicin + Emodin. After 48 h, the cells were fixed and treated with γH2A (CST, USA) for 1 h and then treated with secondary antibody (Alexa-488) for 20 min at RT. The cells were then counterstained DAPI, and then fixed with prolong^®^ diamond antifade mountant (Applied Biosystems, Germany).

### AO/EB (Acridine Orange/Ethidium Bromide) Staining

The BC cells were treated with Emodin for 48 h and then incubated with AO/EB solution for 5 min (Solarbio of Biotechnology, China). The rate of cell death was computed as shown below:

$$Apoptotic\;rate\;(100\%)=\frac{Apoptotic\;cells}{All\;Cells}$$

### Tumor Xenograft Assay and Immunohistochemistry

Mice (nude) experiments were approved by Harbin Medical University Cancer Hospital. Twelve female nude mice (5–6 weeks) weighing ~20 g were obtained from Beijing Charles River (Beijing, China) and randomly divided into two groups (The control and treatment/Emodin group). The animals were kept at the animal house in standard cages and fed on rodent feed and water *ad libitum*. Tumors bodies were injured by 1 × 10^6^ MCF-7 cells in the right flank of mice. The experiment was conducted for 21 days and none of the study animals died. The health and behavior of the mice were monitored after every 3 days. The tumor diameter was measured by a caliper and the tumor tissues were used to test the expression of KI67 by immunohistochemistry.

### Defining the Differentially Expressed Genes and Potential Signaling Pathways Affected by Emodin in MCF-7 Cells

We used GSE111803 and the Student’s t test and fold change to identify the differentially expressed genes (DEGs) in Emodin-treated MCF-7 cells. We compared the expression of the mRNAs from TPM standardized data between the two groups and the significance was set at *p* < 0.05, (|log2FD|>1). The functions and the potential signaling pathways of the DEGs were further explored using the Kyoto Encyclopedia of Genes and Genomes (KEGG) analysis and the Database for Annotation, Visualization, and Integrated Discovery (DAVID) tool.

### Data Analysis

All the data was acquired from at least 3–6 independent experiments and were presented as a mean ± SD. Data from the two groups was assessed by the paired Student’s t test while statistical significance in multiple groups was determined using ANOVA. The *P* < 0.05 was considered as significant.

## Results

### Emodin Inhibits the Growth of BC Cells in a Dosage-Dependent Manner

The viability of BC cells (MCF-7 and MDA-MB-231) in Emodin pressure was interrogated by the CCK-8 assay. Our data showed that Emodin represses the cell viability in a dosage-dependent way (0–500 μM) for 48 h (**Figure 1A**). The Emodin IC_50_ was 90.2 ± 2.1 and 109.1 ± 1.6 μM in MCF-7 cell and MDA-MB-231 cells, respectively. Besides, the AO/EB data demonstrated that at 110 μM, Emodin could induce apoptosis in BC cells (**Figure 1B**). In addition, flow cytometry assays showed that Emodin can induce apoptosis in breast cancer cells (**Figure 1C**).

**Figure 1:** Emodin inhibit BC growth *in vitro*. BC cells were treated with Emodin for 48 h, **(A)** CCK-8 assay showed that Emodin inhibits BC cell growth in a dose-dependent manner. **(B, C)** AO/EB staining and Flow cytometry were used to detect the apoptosis in BC cells. T test. *P < 0.05 vs Control group.

### Emodin Suppress Tumor Growth *In Vivo*

We used nude mice experiments to test the effect of Emodin in tumor growth. The mice were subcutaneously injected with MCF-7 cells in PBS, and Emodin into the flanks of the mice. Compared with the control group, Emodin significantly inhibited tumor growth and decreased tumor weight (**Figure 2A**), as well as KI67 expression (**Figure 2B**). In addition, our data demonstrated that tumor growth was slower in the Emodin group compared to the control group (**Figures 2C, D** **)**. These findings suggested that Emodin suppresses tumor growth *in vivo*.

**Figure 2:** Emodin inhibits tumor growth *in vivo*. **(A)** Tumor morphology. **(B)** The level of KI67 expression in tumor tissues. **(C)** The weight of tumor bodies. **(D)** The volume of tumor bodies. T test. *P < 0.05 vs Control. **P < 0.01 vs Control.

### Emodin Sensitizes BC Cells to Doxorubicin

Next, we investigated the effect of Emodin in BC cells’ susceptibility toward doxorubicin. Treatment of the cells with Emodin (110 μM for 48 h) robustly increased the sensitivity of the BC cells to doxorubicin (**Figures 3A, B** **)**. Interestingly, MCF-7 cells were more sensitive to the combination of Emodin + doxorubicin than the MDA-MB-231 cells. Five μM doxorubicin in combination with 110 μM Emodin inhibited the growth of MCF-7 cells and MDA-MB-231 cells by 21 and 18%, respectively. This data demonstrates that effect of Emodin depends on the genes mediating BC development.

**Figure 3:** Emodin enhances the sensitivity of BC cells to doxorubicin. **(A)** BC cells (MCF-7 and MDA-MB-231) were treated with Emodin and Doxorubicin for 48 h. CCK-8 assay shows that Emodin (110 μM) enhances the sensitivity of MCF-7 cells to Doxorubicin. **(B)** A combination of Emodin (110 μM) and Doxorubicin significantly decreases the growth of MDA-MB-231 cells compared with single Doxorubicin treatment. **P < 0.01, * *P* < 0.05 compare with Doxorubicin group. The analysis was conducted using the Student’s t-test.

### Emodin Stimulates DNA Damage Caused by Doxorubicin in BC Cells

DNA damage is a major mechanism by which doxorubicin acts in BC or TNBC (28–30). To test our hypothesis, γH2A staining was used as a direct way to show shifts in DNA damage and drug resistance in BC cells. We demonstrate that a combination of doxorubicin + Emodin increases the γH2Ax expression compared to either doxorubicin or Emodin treatment alone (**Figures 4A, B** **)**. This finding suggest that Emodin enhanced the effect of doxorubicin by enhancing the DNA damage activities of doxorubicin.

**Figure 4:** Emodin promotes DSB induced by doxorubicin. γH2A staining shows Emodin (110 μM) increases the expression of γh2A and promotes tailing in **(A)** MCF-7 and **(B)** MDA-MB-231 cells as induced by doxorubicin (5 μM). **P < 0.01 vs doxorubicin group. The analysis was conducted using the Student’s t-test.

### Emodin Arrests AKT1 Expression and PI3K-AKT Signaling Pathway in BC

To further investigate the potential mechanisms of action of emodin in inhibiting BC, we used GSE111803 data to identify DEGs after Emodin treat in MCF-7 cells. A total of 158 mRNAs were selected and their expression profile was evaluated from microarray data (p < 0.05, |log2FC|>1). Sixty-eight mRNAs were up-regulated while 90 were down-regulated (**Figure 5A**). Functional enrichment analysis of the DEGs revealed that the PI3K-AKT pathway was significantly enriched (**Figure 5B**).

**Figure 5:** Emodin arrests AKT1 expression and Chemical carcinogenesis signaling pathway in MCF-7 **(A)** The volcanic map of DEGs in GSE111803 data set. **(B)** Pathway enrichment of DEGs.

### Emodin Reduces the Expressions of XRCC1, PARP1, p53, RAD51, and AKT1 Signaling Pathway

Our bioinformatics analysis revealed that Emodin could potentially influence PI3K-AKT pathway (**Figure 3B**). On the other hand, other reports showed AKT1 played an important role in the resistance of BC cells toward doxorubicin (31) (32). Here, we analyzed the expression of AKT1 and DNA damage proteins (XRCC1, PARP1, p53, and RAD51) in BC cells treated with Emodin (110 μM for 48 h). Our data showed that the expression of AKT1 was downregulated by ~0.35-fold in cells treated with Emodin. Similarly, the expression of XRCC1, PARP1, and RAD51 proteins was reduced after treatment with Emodin (**Figures 6A, B** **)**, while p53 protein expression was increased.

**Figure 6:** Emodin down-regulates the expression of AKT1, XRCC1, PARP1, and RAD51. BC cells were treated with Emodin (110 μM), for 48 h. The western blotting data shows that Emodin down-regulates the protein levels of AKT1, XRCC1, p53, PARP1, and RAD51. **(A)** MCF-7 and **(B)** MDA-MB-231. *p < 0.05 vs the control group. The analysis was conducted using the Student’s t-test.

### AKT1 Regulates DNA Damage to Decrease the Cell Viability of BC Cells Toward Emodin

So far, we have established that AKT1 might be mediating the Emodin actions and DNA damage in BC. We successfully overexpressed AKT1 in BC cells (**Figure 7A**) and assayed the cells’ sensitivity to Emodin. Testing the BC cells’ viability in Emodin pressure showed that the cells bearing the overexpressed AKT1 reduced their susceptibility toward Emodin (**Figure 7B**). Besides, γh2A staining also suggested that the down-regulation of AKT1 sensitizes the cells to DNA damage, while up-regulate AKT1 resist the resists the cells to DNA damage, and it is an important occurrence in mediating the efficacy of Emodin in BC treatment (**Figures 7C, D** **)**.

**Figure 7:** BC cells complemented with AKT-1-si or AKT-1-oe regulated to Emodin. **(A)** The expression of AKT1 after treatment with AKT1-siRNA or AKT1 over-expression. **(B)** CCK-8 assay shows the BC cells complemented with AKT1-siRNA or AKT1 over-expression. **(C)** DNA damage assays shows that the BC cells complemented with AKT1-siRNA promote Emodin compared with cells treated with AKT1-siRNA or Emodin alone. **(D)** DNA damage assays shows that the BC cells complemented with AKT1 over-expression resists Emodin compared with cells treated with AKT1-overexpression or Emodin alone. The analysis was conducted using the Student’s t-test. *p* > 0.05, **p < 0.01, *p < 0.05.

## Discussion

Drug resistance threatens the global fight against cancer. In our study, we demonstrate that Emodin does not only inhibit BC cell growth but also sensitizes the BC cells to doxorubicin by acting on AKT1 and regulating DNA damage pathways. Emodin (1, 3, 8-trihydroxy-6-methylanthraquinone) is a natural anthraquinone derivative that isolated from herbs. Emodin has been reported to have a wide spectrum of pharmacological applications, especially hepatoprotective, anti-inflammatory, antibacterial and anti-cancer effects. Evidence shows that Emodin has a tumor-suppressor activity in many cancers (33, 34), especially the intrinsic insensitivity of cancer cells to drugs (34). Our *in vivo* and *vitro* assays showed that Emodin suppresses the cell growth and induces apoptosis in BC cells.

Previous studies have shown that Emodin reverses the colorectal cancer (CRC) resistance toward 5-Fu by downregulating the PI3K/Akt signaling pathway (35). Besides, Wang et al., reported that Emodin could enhance the sensitivity of pancreatic cancer cells to EGFR inhibitors (36). Tong et al. showed Emodin reverses gemcitabine resistance of pancreatic cancer cell lines through inhibition of IKKbeta/NF-κB signaling pathway (37). Bhattacharjee M et al. suggested that combinatorial therapy of thymoquinone and emodin synergistically enhances apoptosis, attenuates cell migration, and reduces stemness efficiently in breast cancer (38). These rose the question that whether emodin could increases the sensitivity of BC to doxorubicin. To investigate this, we evaluated the efficacy of Emodin in the treatment of BC cells and then used γH2A to examine doxorubicin-induced DNA damage in BC cells, with or without Emodin. Our data showed that Emodin increases the sensitivity of BC to doxorubicin. We, further, observe that Doxorubicin causes DNA damage and is a crucial step in inducing cancer cell apoptosis (39–41). To test the DNA damage phenomenon, we used γH2A, a special marker of DNA damage, to stain the cells. The γH2AX staining data showed that Emodin synergizes doxorubicin to induce more DNA damage leading to cell death (**Figure 4**).

To further investigate the potential mechanisms of action of Emodin in BC, we conducted bioinformatics analysis on GSE111803. The functional annotation result showed that PI3K-AKT pathway was significantly enriched (**Figure 5B**). Previous evidence showed that AKT1 plays an important role in the resistance of BC cells toward Doxorubicin (31) (32). Emodin has also been reported to stimulate mixed cell death, augmentation of oxidative stress, DNA damage, and suppression of AKT in cervical and oral squamous carcinoma cell lines (13). AKT1, an important member of the AKT family, accelerates tumorigenesis and has pro-migratory effects (42). We hypothesized that Emodin sensitizes BC toward doxorubicin through AKT1-related pathways. As expected, compared to the control group, Emodin decreased the expression of AKT1 in BC cells. The data showed that AKT1 is an important protein in mediating Emodin’s inhibitory effects on BC cell proliferation. Furthermore, we investigated the Emodin’s effect on DNA damage relate proteins XRCC1 (a scaffold protein that interacts with BER factors), PARP1, RAD51. Our data showed that Emodin decreases the expression of XRCC1 in BC cells as compared to the control group. We also found that Emodin marginally down-regulated the expression of RAD51 in BC cells. Together, these data indicate that Emodin enhances the sensitivity of BC to doxorubicin by suppressing AKT1 and other DNA damage proteins.

Finally, our overexpression assays showed that AKT1 upregulation restores the sensitivity of BC cells toward Doxorubicin treatment, while knockdown AKT1 can promote the DNA damage induced by Doxorubicin, suggesting that AKT1 is a key regulator of DNA damage.

Taken together, our finding showed that Emodin inhibits BC cell proliferation and enhances doxorubicin activity against BC cells by regulating AKT1/PI3K/AKT signaling pathway. Nevertheless, there is need for additional studies to further dissect the mechanism of action of Emodin and its interactions with known anti-cancer agents.

## Data Availability Statement

The original contributions presented in the study are included in the article/**Supplementary Material**. Further inquiries can be directed to the corresponding author.

## Ethics Statement

The animal study was reviewed and approved by Harbin Medical University Cancer Hospital.

## Author Contributions

BL and WC designed the study. XZ, LZ, and WC provided the study materials. BL, XZ, LZ, and WC analyzed and interpreted the data. BL wrote the article. All authors contributed to the article and approved the submitted version.

## Funding

This work was supported by the Scientific Research Project of Heilongjiang Province Health and Family Planning Commission (No. 2018475).

## Conflict of Interest

The authors declare that the research was conducted in the absence of any commercial or financial relationships that could be construed as a potential conflict of interest.
